This article has been retracted.

# An Exploratory Study on the Treatment of Obstructive Apnea-Hypopnea Syndrome by Nasal Cavity Expansion

**DOI:** 10.1155/2021/6926509

**Published:** 2021-11-11

**Authors:** Ling He, Zhijin Lin

**Affiliations:** ^1^Hebei Eye Hospital, Otolaryngology-Head and Neck Surgery, Xingtai 054001, China; ^2^Xingtai People's Hospital, Doctor-Patient Communication Office, Xingtai 054001, China

## Abstract

**Background:**

Respiratory disorder is a disease with a very high incidence, in which obstructive apnea-hypopnea syndrome is the most harmful. It has become a common and frequently occurring disease, which seriously influences the health of the affected population. The pathogenesis of obstructive sleep apnea/hypopnea syndrome (OSAHS) is numerous. With the continuous research on OSAHS disease, it has been found that one of its main pathogeneses is caused by the anatomical characteristics of upper airway obstruction induced during sleep. The narrowing and collapse of any plane can affect the ventilation of the upper respiratory tract. In recent years, with the deepening of research, the importance of the upper respiratory tract obstruction as a source of the disease has attracted increasing attention. Nasal stenosis can cause increased nasal resistance, increased pharyngeal inhalation negative pressure, soft palate collapse, and narrow pharyngeal cavity, resulting in open mouth breathing, which can be the initiating factor of the upper airway obstruction. With the development and popularization of nasal endoscopy technology, domestic and foreign scholars have reported more on the treatment of rhinogenic OSAHS with nasal cavity expansion, but they are different. There is still more controversy; the main controversy centered on the effective rate of surgical treatment and the improvement of objective indicators. Therefore, this study performed individualized nasal cavity expansion for patients with OSAHS who are mainly rhinogenic, from subjective symptoms, objective indicators, and effective rate of surgery. *Methods and Patients*. Conduct research and analysis to provide references for the clinical treatment of such patients. For patients with the obstructive apnea-hypopnea syndrome with nasal congestion, individualized nasal cavity expansion was performed to study the clinical effect of nasal cavity expansion in the treatment of OSAHS. This article mainly screens cases through big data and selects a large hospital in China to perform individualized nasal cavity expansion surgery to treat 43 adult OSAHS patients with nasal congestion.

**Results:**

There are uploaded sleep monitoring, nasal reflex, nasal resistance, and nasal symptoms before and after surgery.

**Conclusion:**

Spirometer examination records, along with apnea-hypopnea index and minimum arterial blood oxygen saturation, the minimum cross-sectional area of the nasal cavity, nasal cavity volume, nasal airway resistance, total nasal respiratory volume, and other information. Also we fill in the nasal obstruction symptom assessment scale, sleepiness scale, and study and analyze the surgical effect of nasal cavity expansion.

## 1. Introduction

The obstructive apnea-hypopnea syndrome refers to the collapse and obstruction of the upper airway during sleep, resulting in apnea and hypopnea. It is usually accompanied by snoring, sleep disturbance, and decreased blood oxygen saturation. This leads to daytime sleepiness, inattention, and other symptoms. It can also lead to multiple-organ and multiple-systems damage such as coronary heart disease, hypertension, and type II diabetes. Apnea refers to the cessation of oral and nasal airflow during sleep, that is, a decrease of 90% or more from the baseline level and a duration of 10 seconds or more. Apnea-hypopnea index refers to the average number of apneas and hypopneas occurring per hour [1]. Types of apnea events: apnea events are divided into three types, namely, (i) obstructive, (ii) central, and (iii) mixed. (i) When obstructive breathing disorder occurs, the patient's chest and abdomen breathing are still present. The diagnosis of obstructive apnea syndrome is based on the patient having snoring during sleep, repeated apneas, accompanied by daytime sleepiness, inattention, mood disorders, and other symptoms. At the same time, multichannel monitoring, apnea-hypopnea index (AHI) is greater than or equal to 5 times an hour. When obstructive respiratory events are the main cause, it can be diagnosed as OSAHS. The incidence in men is higher than that in women. With the aging of the population and the increase in obesity, the incidence is increasing year by year [2–4]. With people's attention to the source effects of upper respiratory tract obstructive diseases, the harm of OSAHS has been increasingly recognized [5]. It is often complicated by hypertension in middle-aged and elderly people, and the symptoms of hypoxia when blood pressure is increased. It is closely related to the severity of sleep-disordered breathing [6]. In addition, OSAHS is also an independent risk factor for coronary heart disease. Relevant studies have shown that OSAHS can increase the morbidity and mortality of coronary heart disease. Arrhythmia caused by OSAHS is one of the main causes of nocturnal death [7]. OSAHS is also closely related to the occurrence of type 2 diabetes and can lead to a decline in patients' cognitive function and even mental disorders [8, 9]. With the in-depth study of OSAHS, it is found that the pathogenesis of OSAHS is mainly the narrowing of the upper airway anatomical plane, that is, the partial or complete narrowing and collapse of the airway caused by the obstruction of different planes of the upper airway during sleep. In addition, it also includes pathophysiological mechanisms such as insufficient upper airway dilator response, high loop gain, and low arousal threshold during sleep [10]. With the analysis of anatomical factors on the plane of upper airway stenosis, nasal congestion caused by nasal cavity stenosis may become the initiating factor of upper airway obstruction. Nasal cavity expansion technology can correct nasal anatomy abnormalities through nasal endoscopic surgery, which can improve nasal ventilation and reduce nasal resistance; its core is to increase the effective ventilation volume of the nasal cavity and reduce the anterior upper airway resistance, thereby preventing or improving the collapse of the pharyngeal cavity. It is a surgical technique for the treatment of rhinogenic OSAHS [11], as shown in Figure 1.

In the past, the evaluation of nasal congestion symptoms has mainly relied on the subjective feelings of patients and the estimation of the patient's nasal ventilation through nasal imaging examinations. There is no objective basis, and the patient's subjective feelings are often inconsistent with the actual nasal cavity structure abnormalities. The individual differences of patients and the influence of psychological factors and the existence of nasal menstrual cycle need to objectively quantify the clinical subjective symptoms of nasal obstruction. It is combined with effective auxiliary examinations for comprehensive analysis, which can not only effectively guide clinical work, but also determine the indications for surgery, and can provide an objective reference and objective basis for the prognosis and evaluation of the treatment effect. In recent years, with the continuous advancement of medical engineering technology and the continuous research on the physiological functions of the nasal cavity, the nasal function diagnosis system composed of rhino acoustic reflex, nasal resistance meter, and nasal breath meter has gradually matured. It is been applied in clinical practice, providing clinicians with nasal ventilation function as a basis for objective judgment. Therefore, we incorporate the objective data collected with big data into the objective evaluation of nasal congestion symptoms in patients with rhinogenic OSAHS. Although there are many reports on nasal cavity expansion for the treatment of rhinogenic OSAHS, detailed subjective and objective assessment of nasal congestion and lethargy before and after surgery, a summary of detailed surgical methods, and compliance with continuous positive airway pressure (CPAP) treatment after surgery, there are relatively few comprehensive reports on the improvement of sexual performance and the analysis of different degrees of OSAHS patients among groups. Therefore, through big data screening, we conducted a comprehensive study on nasal cavity expansion surgery to treat rhinogenic OSAHS patients, evaluated and compared various correlation checks, and discussed OSAHS in groups according to the AHI value. We analyzed whether the objective effectiveness of each group was improved after the operation and the degree of improvement, to explore whether nasal cavity expansion can improve the compliance of CPAP therapy and to study the clinical effects of nasal cavity expansion surgery in the treatment of OSAHS and provide references for clinical treatment of such OSAHS patients.

The major contributions of this paper are as follows:

1. This paper proposes the treatment of OSAHS through both nonsurgical and surgical treatments, as well as its related latest treatment suggestions, and the latest treatment methods that may be applied to the clinic.
2. Methods related to the treatment of OSAHS patients are discussed, including drug therapy, CPAP method, nasal surgery, oral appliance, uvulopalatopharyngoplasty (UPPP), and surgery at the bone level.
3. For the treatment of OSAHS patients, CPAP treatment was performed before the operation. The VAS score records the patient's acceptance of CPAP treatment.
4. The efficacy of the treatment used for OSAHS patients is determined.
5. Surgical methods used for OSAHS patients are as follows. All patients in the group underwent individualized nasal cavity expansion surgery under nasal endoscopy, including correction of nasal septum deviation. All patients after correction of nasal septum were subjected to continuous penetration suture of the (i) nasal septum, (ii) selective inferior turbinate surgery, (iii) selective middle turbinate surgery, and (iv) optional bilateral symmetrical opening of the middle nasal passages and sinuses.
6. Postoperative treatments are discussed for the patients before the surgery.
7. The efficacy of surgery is discussed for OSAHS patients. The results show that no complications occurred after endoscopic nasal cavity expansion in all patients.

The outline of this paper is given as follows.

In section 2, Related Work, the methods related to the treatment of OSAHS patients are discussed.

In section 3, Methods, different patients with OSAHS, methods used for the treatment of patients using the CPAP, the efficacy of the treatment used, the surgical methods used for its treatment, and the postoperative treatments are discussed.

In section 4, Experiments and Discussion, the patient's clinical data are analyzed and divided into three groups: mild, moderate, and severe, according to the preoperative PSG monitoring results, statistics of patients' operation, the surgical curative effect of patients, and analysis of CPAP treatment results.

In section 5, Conclusions, a detailed comparative analysis of various related indicators before and after the operation of OSAHS patients with nasal congestion through big data research is discussed.

## 2. Related Work

In recent years, the incidence of OSAHS has increased year by year with the increasing aging of the population and the increase in obesity [12, 13]. In addition, the etiology and pathogenesis of OSAHS are complex and individualized. There are many clinical treatment methods for OSAHS, including behavioral intervention, drug therapy, device therapy, and surgical treatment. Among them, CPAP therapy and oral treatment are the most widely implemented. Therefore, multidisciplinary comprehensive treatment should be used in the clinic according to the individual characteristics of the patient, and the optimal treatment plan should be selected for the patient. This article comprehensively introduces the treatment of OSAHS through both nonsurgical and surgical treatments, as well as its related latest treatment suggestions, and the latest treatment methods that may be applied to the clinic.

Following are the methods related to the treatment of OSAHS.

1. Treatment of OSAHS patients by drug therapy: Drug therapy is mostly adjuvant therapy of OSAHS. In a randomized controlled study of traditional Chinese medicine, it was shown that the addition of phlegm-removing decoction can reduce the oxidative stress and inflammatory response of patients with OSAHS, thereby alleviating their clinical symptoms [14]. In recent years, the treatment of OSAHS by western medicine has been gradually applied to the clinic. Acetazolamide can stimulate respiratory excitement through metabolic acidosis. In a report of 13 patients with OSAHS taking medication for a week, it was pointed out that its effect can reduce the loop gain by 40% or so, AHI halved [15]. In addition, eszopiclone treatment of OSAHS has also been reported such that it is mainly suitable for patients with low arousal threshold and good pharyngeal muscle activity. After treatment, its AHI value can be significantly reduced [16]. The OSAHS is further classified by phenotype, and targeted drug treatment based on the individualized phenotype of OSAHS patients is still the direction of further research [17]. However, in the foreseeable future, CPAP will still be the gold standard therapy for the treatment of OSAHS.
2. Treatment of OSAHS patients by CPAP: At present, CPAP therapy is still the first-line treatment for OSAHS, especially for moderate to severe patients. Several rigorous clinical trials on the efficacy of CPAP treatment have shown that the effect is good, which can significantly improve the patient's daytime sleepiness and quality of life. It can also reduce the incidence of systemic chronic diseases, such as hypertension and cardiovascular disease, and even reduce chronic diseases. Mortality may result from the acute onset of the disease [18–20]. However, many patients with CPAP treatment cannot tolerate or have a weak subjective willingness, and the degree of acceptance is not high. This is mostly because the continuous pressure of CPAP treatment causes respiratory discomfort and dry nose in patients. Therefore, it is more important to choose the appropriate treatment pressure. Titration is critical to the compliance and efficacy of patients with subsequent CPAP therapy [21]. At present, the CPAP technology itself has made many improvements including the diversification of ventilation modes, pipe heating, and humidification, as well as the closure and comfort of the mask, but the degree of improvement in patient compliance is still limited.
3. Treatment of OSAHS patients by the oral appliance: The oral appliance is one of the commonly used conservative treatment options for the treatment of OSAHS. Its therapeutic value has received more and more clinical attention in recent years [22]. At present, the common types of oral appliances are divided into three types: (i) soft palate lifting device, (ii) tongue forward device, and (iii) lower collar forward device. One of the most commonly used is the lower collar forward device. The treatment principle is to move the mandible forward or downward, and the tongue moves forward to widen the upper airway space and increase its stability.
4. Treatment of OSAHS patients by nasal surgery: Nasal surgery is mainly for patients with rhinogenic OSAHS. The surgical methods mainly include three-line nasal septum reduction plasty, selective middle and inferior turbinate surgery, and selective bilateral middle nasal passage and sinus symmetry opening surgery. To correct the abnormal structure of the nasal cavity, volume expansion and nasal surgery can significantly improve patients' daytime sleepiness and nasal congestion symptoms, but there is no significant improvement in postoperative AHI. Nevertheless, domestic and foreign scholars have reported that although AHI has not improved significantly, the quality of life of patients after surgery has been significantly improved, and the expected results before surgery can be achieved [23, 24].
5. Treatment of OSAHS patients by uvulopalatopharyngoplasty (UPPP): Surgery at the velopharyngeal level includes uvulopalatopharyngoplasty (UPPP) and its modified UPPP, as well as hard palate truncation and soft palate advancement. Traditional UPPP surgery has been continuously improved since 1981 and has gradually developed into a commonly used surgical procedure for the treatment of OSAHS [25]: surgical removal of the narrow uvula, part of the soft palate, and bilateral tonsils. However, there are complications such as pharyngeal hemorrhage, nasopharyngeal reflux, and postoperative acute airway obstruction. The success rate of UPPP alone is only 40% [26]. Laser-assisted uvulopalatoplasty (LAUP), soft palate radiofrequency ablation, operation is to reduce the abnormal breathing caused by the vibration and blockage of the soft tissue of the soft palate by reducing the soft tissue of the uvula and palatal sail. LAUP surgery can improve the compliance of patients with continuous positive airway pressure therapy (CPAP), but there are different reports on whether it can reduce AHI [27].
6. Treatment of OSAHS patients by surgery at the bony level: Surgery at the bony level of the oculus mainly includes the advancement of the upper and lower collar bones and the treatment of OSAHS by expanding the volume of the bony airway. The therapeutic effect of this type of surgery on OSAHS is comparable to that of CPAP [28]. A meta-analysis also pointed out that osteoarthritis can be used as a reoperation option for most patients with high residual AHI after the failure of OSAHS surgery [29], given in Table 1.

## 3. Methods

In this section, in the research materials, different patients with OSAHS, methods used for the treatment of patients using the CPAP, the efficacy of the treatment used, the surgical methods used for its treatment, and the postoperative treatments used are discussed below.

### 3.1. Research Material

1. The study subjects selected 43 adult OSAHS patients who were hospitalized in a large hospital in China in July 2019 and underwent individualized nasal cavity expansion surgery, including 39 males and 4 females, with an average age of 40.8 ± 8.6 years. (i) Enrollment criteria are having OSAHS symptoms: sleep at night, intermittent apnea, daytime sleepiness, inattention, nasal congestion, etc. In hospital records, PSG monitors overnight sleep, diagnosed as OSAHS, and AHI is greater than or equal to 5 times per hour, ear and nose laryngology examination. Electronic laryngoscope combined with Muller test, upper respiratory tract three-dimensional CT reconstruction, confirmed that the anatomical structure of the nose was abnormal, with or without oropharyngeal plane stenosis but no throat and throat cavity plane stenosis. The symptoms of nasal congestion did not improve after conservative treatment with drugs. (ii) Exclusion criteria: exclude chronic sinusitis with or without nasal polyps, nasal trauma, nasal benign and malignant tumors, etc.; patients with obvious velopharyngeal stenosis due to tonsil hypertrophy; those with a history of the nasal cavity and sinus surgery; those with endocrine diseases; OSAHS patients, such as acromegaly and hypothyroidism; and patients with a history of mental illness.
2. Main screening and recording parameters are minimum cross-sectional area of the nasal cavity, nasal cavity volume, nasal resistance value, total nasal respiratory volume.

### 3.2. Research Method

All patients recorded their age, gender, and BMI index; see Table 2. CPAP treatment was performed before the operation. The VAS score records the patient's acceptance of CPAP treatment. The score is 0–10 points. The higher the value is, the more difficult it is to receive CPAP treatment. Manual pressure titration records the average effective treatment pressure. For score by Epworth Sleepiness Scale, see Table 3 for details, score the sleepiness symptoms of patients. For filling in the NOSE scale, see Table 4, simulating the specific records of nasal congestion in patients with rhinogenic OSAHS. Screening the patient's nasal acoustic reflex, nasal resistance, and nasal breath meter recording data, as well as NMCA, NCV, and NAR, *V*_T_ data represent objective evaluation indicators for nasal congestion. Among them, NCV is the 0-7 cm nasal ventilation volume of the nasal cavity, and NAR is the total double-nasal inspiratory image. Resistance, *V*_T,_ is the total respiratory volume of nasal breathing. In addition, the preoperative AHI and LSaO_2_ data recorded by the uploaded PSG are divided into mild, moderate, and severe according to the diagnosis basis and curative effect evaluation criteria of the Chinese Medical Association. Recheck the above items 3 months after the operation. The uncured patients will be treated with CPAP again and the VAS score and the average effective treatment pressure of CPAP treatment will be recorded. The scoring standard is 0–10 points. The higher the score is, the more difficult it is to receive CPAP treatment.

### 3.3. Efficacy Judgment

With AHI as the standard, the therapeutic effect was determined by the 2009 obstructive apnea-hypopnea syndrome diagnosis and surgical treatment guidelines. The patient's subjective symptoms and changes in hypoxemia were also considered in the determination: (1) cure AHI less than 5 times per hour; (2) significantly effective: AHI less than 20 times per hour and a reduction greater than or equal to 50%; and (3) effective: AHI reduction greater than or equal to 50%.

### 3.4. Surgical Method

According to all statistical objects screened by big data, their surgical methods are as follows. All patients in the group underwent individualized nasal cavity expansion surgery under nasal endoscopy, including correction of nasal septum deviation. All patients after correction of nasal septum were subjected to continuous penetration suture of the (i) nasal septum, (ii) selective inferior turbinate surgery, and (iii) selective middle turbinate surgery, and (iv) optional bilateral symmetrical opening of the middle nasal passages and sinuses. All patients were treated with general anesthesia under tracheal intubation after excluding the contraindications of the operation. During the operation, the position was the supine position with head high and feet low about 15°, and the bilateral nasal cavity was constricted with normal saline and epinephrine cotton pads during the operation.

(1) Correction of nasal septum deflection: It is suitable for patients with nasal septum deflection which leads to limited nasal ventilation or airflow disturbances and even affects the drainage of the middle nasal passage. The second-line nasal septum reduction plasty was performed in all operations. The incision was made at the junction of the skin and mucosa of the nasal vestibule with an L-shaped incision and extended to the outside of the nasal base. The mucosa and mucochondrium were incised and peeled off under the mucochondrium. Dissection of the mucochondrium was performed under direct endoscopy. The dissection range included the lower end of the nasal septal cartilage and its connection with the maxillary palatine process and the vomer, the vertical plate of the ethmoid bone, and the upper posterior part of the vomer. Three core areas of tension formation are revealed, including the end of the nasal septal cartilage, the junction of the nasal septal cartilage, and the vertical plate of the ethmoid. During the operation, three linear bone strips were bitten out according to the need for correction of nasal septum deviation. Form the nasal septal cartilage top connection; separate the left and right sides; free the front, back, and bottom three sides; and classify and remove the spinous processes up and down. For those with obvious high deflection, rongeurs can be used to clamp the ethmoid vertical plate to make it fracture without being removed. Pay attention to protecting the connection area of the nasal bone, nasal septal cartilage, ethmoid vertical plate, and nasal dorsal cartilage to prevent the back of the nose from collapsing. Causes of nasal congestion: nasal congestion is caused by the deflection of the nasal valve area, it is the narrowest part of the nasal cavity, and the nasal resistance is higher, which is likely to cause more serious OSAHS. Simply removing the tension curve or simply removing the cartilage strips at the end of the nasal septum cartilage is often not enough. It is necessary to separate the end of the nasal septum cartilage from the inner foot of the alar cartilage and remove part of the end of the nasal septum cartilage in a wedge shape to correct the dislocation or subluxation of the nasal columella. After remodeling, it is stitched through. If the combined nasal septal cartilage has deviated, you can cut the cartilage on the convex surface several times to reduce its tension. If it is a simple crista bony deviation, a longitudinal incision can be made on the surface of the deviated bone to protect the integrity of the contralateral mucosa by removing the cristae and reducing the mucosa.
(2) Continuous nasal septum suture: After correction of nasal septum deviation, we routinely perform continuous nasal septum suture, using absorbable suture with needles, first intermittently suture the nasal septum incision with 3 stitches, and finally leave a single tail thread to tie the suture with the through suture. Fix then tie the end of the suture needle, hold the end of the suture with the needle holder longitudinally, enter through the left nasal cavity, perform the first stitch through the upper part of the middle turbinate, and suture to the right nasal cavity and then on the right side of the nasal septum. The lower part of the nasal cavity is inserted into the left nasal cavity, and then the continuous suture in the shape of “bow” is performed in this way. When the nasal septal cartilage is close to the front end of the nasal septum, ensure that the last two sutures are aimed at the remaining nasal septal cartilage during the operation. A penetrating suture is used to shape the middle of the nasal septum, and, finally, the penetrating suture and the indwelling suture at the front end of the nasal septum are knotted and fixed at the bottom of the left nasal vestibule. After the operation, only absorbent cotton can be used for packing.
  1. Selective inferior turbinate surgery: According to the patient's specific disease conditions, there are three types of surgery. (i) The first is the partial submucosal resection of the inferior turbinate, which is mainly for patients with inferior turbinate bone hyperplasia. Local infiltration anesthesia is applied along the bottom of the inferior turbinate and a longitudinal incision is made to protect the normal inferior turbinate mucosa and remove the hyperplastic bone. Move out and reset the inferior turbinate. (ii) The second is the external transfer of inferior turbinate fractures. It is suitable for patients with mild hypertrophy of the inferior turbinate. The bone mass of the inferior turbinate is fractured by the stripper and fixed externally to widen the total nasal passage area. (iii) The third type is plasma submucosal ablation of the inferior turbinate, which is suitable for the inferior turbinate mucosa and is not thick bones. A needle-like plasma knife is used to perforate the front end of the inferior turbinate, and the inferior turbinate mucosa is ablated from front to back. Absorbent cotton was used to fill and shape the inferior turbinate after the operation. In the case of submucosal resection of the inferior turbinate, absorbent cotton can be cut longitudinally during packing and placed in the common nasal passage and lower nasal passage, respectively, to shape and fix the inferior turbinate.
  2. Selective middle turbinate surgery: According to the patient's specific disease conditions, there are three types of surgery. (i) The first is the partial submucosal resection of the middle turbinate, which is mainly for patients with bone hyperplasia of the middle turbinate. Local infiltration anesthesia is applied along the free edge of the middle turbinate and a longitudinal incision is made. (ii) Repositioning the middle turbinate inward; the second is the internal fixation of the middle turbinate, which is suitable for patients with mild hypertrophy of the middle turbinate or reverse curvature of the middle turbinate. Use the stripper to directly move the middle turbinate inward with light pressure to widen the middle nasal passage. (iii) The third type is the partial resection of the middle turbinate, which is mainly suitable for patients with the middle turbinate bubble. Use a sharp knife to puncture the middle turbinate air chamber, resect the outer wall of the air chamber in a sagittal position, retain the inner wall, and trim the margin and move it inward and fix it. The turbinate fully widens the middle nasal passage. Here for the scope of middle turbinate resection, we generally control the lower edge of the middle turbinate higher than the upper edge of the inferior turbinate, and the front edge of the middle turbinate is located behind the frontal process of the maxillary, and the distance is generally greater than 5 mm. This can effectively maintain a good shape of the middle turbinate, meet functional requirements, ensure drainage of the middle nasal passage, and prevent postoperative adhesions. After the operation, absorbent cotton was routinely placed on the outside of the middle turbinate for packing to ensure the shape of the middle turbinate.
  3. Selective bilateral symmetrical opening of the middle nasal passages and sinuses: for the uncinate hypertrophy or gasification and middle nasal passages stenosis, after treatment according to the shape of the middle turbinate, bilateral uncinate resection is performed, and the scope of the resection of the uncinate process is as follows: keep a little at the upper end, and excise the lower end to expose the ostium of the maxillary sinus. If there is still a possibility of poor maxillary sinus drainage after uncinate process resection, bilateral maxillary sinuses should be opened symmetrically. For those with overdeveloped ethmoid vesicles or the formation of Haller air cells and nasal mound air cells, anterior sieve should be performed opening the sinuses and opening the frontal and maxillary sinuses as appropriate to avoid occlusion of the sinus. For patients with nasal cavity stenosis, due to the gasification of the maxillary sinus, the nasolacrimal crypt approach is used to protect the nasolacrimal duct to remove the inferior turbinate bone and remove the targeted part. The bone of the inner wall of the maxillary sinus is combined with the middle nasal passage to remove the uncinate process. The bilateral maxillary sinuses are opened symmetrically, and the inferior turbinate and outer wall of the nasal cavity is moved outward; the inferior turbinate is pushed into the upper mandibular sinus cavity to expand the inherent nasal cavity area.

### 3.5. Postoperative Treatment

According to the postoperative treatment records of the screening subjects recorded by the hospital, nasal spray with seawater was performed 24 hours after the operation, and nasal cavity washing was performed 48 hours later. The nasal cavity was observed for bleeding and infection under anterior rhinoscopy, and the total was cleaned on the third day after the operation. Nasal secretions were discharged from the hospital on the 4th day after surgery and were treated with nasal spray hormones and oral mucus excretion agents. After 7–10 days of the operation, the nasal cavity packing was removed by the dressing change of the nasal endoscopy, and the nasal cavity suture was removed for the patients with nasal septum correction. Routine nasal endoscopy was performed 4 weeks, 8 weeks, and 12 weeks after surgery to clean the nasal cavity and prevent intraoperative adhesions. Three months after the operation, recheck and fill in the NOSE scale and ESS scale to record scores; recheck PSG to record AHI and LSaO_2_; recheck nasal reflex, nasal resistance, and nasal breath meter examination; and record NMCA, NCV, NAR, and *V*_T_. CPAP treatment was performed on uncured patients, and the VAS score of CPAP treatment was recorded and the average effective treatment pressure was recorded by pressure titration.

## 4. Experiments and Discussion

In the experiments and discussion section, the patient's clinical data are analyzed and divided into three groups mild, moderate, and severe according to the preoperative PSG monitoring results. Statistics of patients' operation, the surgical curative effect of patients, and analysis of CPAP treatment results are discussed.

### 4.1. Analysis of Patient Clinical Data

All 43 patients screened based on big data were grouped according to the preoperative PSG monitoring results according to the AHI value and divided into three groups: mild, moderate, and severe, including 16 cases in the mild group, 14 males and 2 females; 13 cases in the moderate group, 11 males and 2 females; 14 patients in the severe group, all males. The ages between the three groups were mild: 34.7 ± 6.2, moderate: 41.2 ± 7.2, and severe: 47.8 ± 6.5. BMI between the three groups were, respectively, mild: 22.5 ± 1.7 kg/m^2^, moderate: 24.8 ± 2.3 kg/m^2^, and severe: 27.6 ± 2.7 kg/m^2^. A single factor is used for the comparison of age and BMI index among the three groups for the analysis of variance; see Table 5 and Figure 2 for age and see Table 6 and Figure 3 for the BMI index. The results of the single-factor analysis of variance for the age of the three groups of patients were *F* = 14.26, *P* < 0.05, and the result of the BMI index single-factor analysis of variance was *F* = 20.39, *P* < 0.05, indicating the severity of OSAHS patients. There is a tendency to increase with age and the severity of OSAHS increases with the increase in BMI.

### 4.2. Statistics of Patient Operations

All patients underwent nasal septum deflection correction in 39 cases; middle turbinate submucosal partial bone resection was performed in 6 cases, middle turbinate internal fixation was performed in 30 cases, and middle turbinate was partially resected in 9 cases; bilateral inferior turbinate was performed in 9 cases. There were 29 cases of partial submucosal resection, 9 cases of unilateral partial submucosal resection of the inferior turbinate and 7 cases of inferior turbinate fractures.

### 4.3. The Effect of Surgery

According to the record results shown by big data, among the 43 samples, 7 cases were cured, 8 cases were markedly effective, and 3 cases were effective, including 5 cases of mild OSAHS cured, 5 cases of marked effect, 2 cases of moderate OSAHS cured, 3 cases of marked effect, and severe OSAHS effect in 3 cases. The overall effective rate is 41.9%, as shown in Figure 4. No complications occurred after endoscopic nasal cavity expansion in all patients.

### 4.4. Analysis of CPAP Treatment Results

After nasal cavity expansion, the NOSE score and ESS score of all patients were significantly decreased, and the subjective nasal congestion and drowsiness symptoms were significantly alleviated. The objective indicators of NMCA, NCV, *V*_T_ increased significantly, and the NAR decreased significantly. Indicating that the patient's nasal cavity was significantly more spacious than before surgery and ventilation increased; see Table 7 for details. Compared with preoperative patients, the VAS scores of CPAP treatment and the average effective treatment pressure of CPAP treatment were significantly reduced, and the average *P* < 0.05. According to the efficacy evaluation standard of the Chinese Medical Association, in this study, after the treatment of nasal cavity expansion surgery, the AHI of the mild and intermediate OSAHS patients decreased, and the LSaO_2_ increased, *P* < 0.05. Although the AHI of the severe group OSAHS patients decreased, the LSaO_2_ increased, *P* > 0.05; see Table 8.

## 5. Conclusions

This study conducted a detailed comparative analysis of various related indicators before and after the operation of OSAHS patients with nasal congestion through big data research. By comparing the preoperative and postoperative results and combining the subjective NOSE scores filled in by the patients at the time, the operation of such OSAHS patients was carried out. The postnasal congestion was analyzed subjectively and objectively. A relatively novel surgical method of external movement of the outer wall of the nasal cavity and continuous suture of the nasal septum was proposed. The different treatments of the inferior turbinate and the surgical treatment and indications of the bilateral symmetrical opening of the sinuses are summarized. In addition, the light, moderate, and heavy groups of OSAHS are discussed through the PSG examination records and compared with the preoperative and postoperative AHI, LSaO_2,_ and the patient's filling in at the time. The subjective ESS score of the nasal cavity was discussed, and the different effects between the groups after nasal cavity expansion were discussed. The reasons for the different effects between the groups were explained, indicating that some moderate and severe OSAHS patients still need multilevel comprehensive treatment. The above are all clinical work, providing more meaningful reference data. In addition, through the questionnaires filled out by patients, it is found that the patient's subjective acceptance of CPAP treatment and objective CPAP effective treatment pressure are summarized in two aspects. Nasal cavity expansion surgery can improve compliance with CPAP treatment. However, this study also has some shortcomings, such as the relatively short research time and the small number of research samples. In addition, the inconsistency between subjective symptoms and objective indicators requires further in-depth research. Therefore, the research results of this paper still need follow-up long-term field visits and further observation and research.

## Figures and Tables

**Figure 1:** Nasal cavity expansion.

**Figure 2:** The number and age distribution of the three groups of OSAHS patients.

**Figure 3:** The number of OSAHS patients in each group and BIM index in the three groups.

**Figure 4:** Statistics chart of surgical curative effect of patients with different degrees.

**Table 1:** Symbol description.

English abbreviations	English full name
OSAHS	Obstructive apnea-hypopnea syndrome
AHI	Apnea-hypopnea index
CPAP	Continuous positive airway pressure
LAUP	Laser-assisted uvuloplasty
UPPP	Uvulopalatopharyngoplasty
ESS	Epworth sleep scale
PSG	Polysomnogram
VAS	Visual analogue scale
NMCA	The nasal minimum cross-sectional area
NCV	Nasal cavity volume
NAR	Nasal airway resistance
*V*_T_	Nasal total volume
LSaO_2_	Lowest arterial oxygen saturation

**Table 2:** BMI (kg/m^2^) guideline.

BMI classification	WTO standards	China standard	Disease risk
Thin	<18.5	<18.5	Low
Normal	18.5∼24.9	18.5∼23.9	Average
Overweight	≥25	≥24	Increase
Little obesity	25.0∼29.9	24.0∼26.9	Increase
Obesity	30.0∼34.9	27∼29.9	Moderate increase
Severe obesity	35.0∼39.9	≥30	Severe increase

**Table 3:** Epworth Sleepiness Scale.

Item	Never drowsy	Slightly drowsy	Moderately drowsy	Severe drowsy
Reading book	0	1	2	3
Watching TV	0	1	2	3
Sit still	0	1	2	3
One hour by car	0	1	2	3
Lunch break	0	1	2	3
Sit and talk	0	1	2	3
Lunch	0	1	2	3

Tips: >6 means drowsy, >11 means over drowsy, and >16 means dangerous drowsy.

**Table 4:** The NOSE scale for the evaluation of nasal obstruction symptoms.

Item	Not	Slightly	Moderately	Serious	Dangerous
Nose airtight	0	1	2	3	4
Nose stuffy	0	1	2	3	4
Insomnia	0	1	2	3	4
Movement difficulties	0	1	2	3	4

**Table 5:** Statistical distribution of three groups of OSAHS patients at different ages.

Grouping	Number	Age	*F*	*P*
Mild	16	34.7 ± 6.2	14.26	<0.05
Moderate	13	41.2 ± 7.2		
Severe	14	47.8 ± 6.5		

**Table 6:** One-way variance of BIM in three groups of OSAHS patients.

Grouping	Cases number	Age	*F*	*P*
Mild	16	34.7 ± 6.2	14.26	<0.05
Moderate	13	41.2 ± 7.2		
Severe	14	47.8 ± 6.5		

**Table 7:** Congestion and lethargy before and after surgery.

Check index	Before surgery	After surgery	T	*P*
NOSE	12.4 ± 2.86	4.5 ± 1.77	19.83	<0.001
ESS	12.7 ± 2.21	7.6 ± 2.14	23.69	<0.001
NMCA (cm^2^)	0.5 ± 0.11	1.5 ± 0.26	−41.18	<0.001
NCV (cm^3^)	8.9 ± 0.83	18.2 ± 3.26	−19.56	<0.001
NAR (kPa•s/L)	0.5 ± 0.04	0.2 ± .0.03	50.79	<0.001
*V*_T_ (L)	5.2 ± 0.47	8.7 ± 1.54	−18.67	<0.001

**Table 8:** Comparison of AHI and LSaO_2_ of patients before and after surgery.

Grouping	Check index	Before surgery	After surgery	*t*	*P*
Mild	AHI	10.8 ± 2.7	6.3 ± 2.34	6.92	<0.001
	LSaO_2_	76.4 ± 2.6	82.0 ± 2.80	−12.45	<0.001

Moderate	AHI	24.4 ± 4.4	17.4 ± 6.51	6.03	<0.001
	LSaO_2_	70.9 ± 3.2	73.9 ± 3.29	−8.88	<0.001

Severe	AHI	055.4 ± 14.5	53.4 ± .19.8	0.81	0.436
	LSaO_2_	65.9 ± 4.62	66.9 ± 3.30	−1.33	0.210

## Data Availability

The datasets used and analyzed during the current study are available from the corresponding author upon reasonable request.
